# KL-FGF23-VD Axis in Improving Late-Onset Alzheimer's Disease by Modulating IKK/NF-*κ*B Signal Pathway

This article has been retracted.

**DOI:** 10.1155/2022/3100621

**Published:** 2022-09-09

**Authors:** Yingying Cai, Jiali Hu, Mingjie He

**Affiliations:** ^1^Department of Geriatrics, The First Affiliated Hospital of Chengdu Medical College, Chengdu 610500, China; ^2^Medical Department, The First Affiliated Hospital of Chengdu Medical College, Chengdu 610500, China

## Abstract

**Materials and Methods:**

LOAD rats and A*β* microglia were constructed by using A*β*_1-40_ and IBO mixture. The effect of KL-FGF23-VD axis on LOAD was investigated by transfecting overexpressing and interfering with KL gene adenovirus, and IKK-16 was added to A*β* microglia to explore the effect of KL-FGF23-VD axis on regulation of IKK/NF-*κ*B signaling pathway.

**Results:**

The results showed that, in KL-OE group, FGF23 was decreased in the hippocampus of LOAD rats compared with control and KL-si, and the trend was opposite in the KL-si group. The KL-FGF23-VD axis can alleviate inflammatory response, reduce the deposition of A*β*, and inhibit activation of the NF-*κ*B pathway and neuron apoptosis in brain tissue of LOAD rats. In A*β* microglia, the expression of KL-FGF23-VD axis was consistent with animal experiments. The KL-FGF23-VD axis can inhibit the expression of A*β* microglia inflammatory factors and the activation of microglia and NF-*κ*B pathway. Meanwhile, IKK expression was decreased in KL-OE group compared with KL-si and Control. In the IKK-16 addition group, the ability of KL-FGF23-VD axis to inhibit the activation of microglia and NF-*κ*B pathway was enhanced.

**Conclusions:**

These findings suggest a potential role of the KL-FGF23-VD axis in AD treatment by regulating the IKK/NF-*κ*B pathway.

## 1. Introduction

Alzheimer's disease (AD) was first reported in 1906 by Alois Alzheimer, a clinical psychiatrist and neuroanatomist in Tübingen. The report describes a 50-year-old woman with clinical features of progressive sleep, memory impairment, aggression, and delirium, with marked plaques and neurofibrillary tangles in her brain histology [1]. This disease is progressive and neurodegenerative, leading to damage including physical, emotional, and cognitive functions. Late-onset Alzheimer's disease (LOAD) is a degenerative disease of the central nervous system, which is characterized by progressive impairment of cognition and behavior after 65 years old.

The main pathological manifestations of Alzheimer's disease in the brain tissue are senile plaques caused by excessive deposition of beta-amyloid protein (A*β*), hyperphosphorylated neurofibrillary tangles (NFTs) caused by hyperphosphorylation of Tau protein, neuronal degeneration and death, etc. Its etiology and pathogenesis are still unknown, but most studies indicate that neuroinflammatory mechanisms play an important role in LOAD [2, 3]. 99% of patients belong to sporadic AD whose main pathological mechanism is that A*β* is abnormally cleavage and metabolized due to some factors including gene mutation, neurotransmitter disorder, oxidative stress, free radical damage, and inflammatory response, which result in the removal impairment of A*β* and thus lead to excessive deposition of A*β* [4, 5]. Excessive A*β* has strong self-aggregation, is easy to form *β*-sheet structure and further aggregation to form senile plaques, activates microglia, promotes inflammatory response, induces abnormal phosphorylation of tau protein and NFT, and damages synapses and neurons, eventually leading to neuronal apoptosis and dementia [6–8].

Klotho gene (KL) knockout mice exhibited symptoms of aging (including cognitive decline), while their life span was prolonged by 20–30% after overexpression in mice. This suggests that KL gene may be an age-suppressing gene [9]. KL may also be a gene related to human elder age and central nervous system function. KL is mainly distributed in the cerebellar Purkinje fibers and choroid plexus of rat brains. It is also observed in gray matter (including the cortex and hippocampus) and can be detected in cerebrospinal fluid, blood, and gray matter [10, 11]. Studies have confirmed the effect of KL in protecting hippocampal neurons, and KL level in plasma is correlated with the cognitive function of the elderly without dementia [12–14]. KL gene polymorphisms are associated with cognitive function in 90–100-year-olds [15]. Moreover, it has been reported that KL gene can improve the cognitive ability of dementia mice and reduce mortality [16, 17].

Fibroblast growth factor-23 (FGF23) serves as an important endocrine factor secreted by osteoblasts, which can regulate the metabolism of calcium, phosphorus, and vitamin D (VD) in vivo. KL can block the expression of FGF23, and the secretion of FGF23 increased in KL knockout mice [18]. Drew et al. found that there was a correlation between FGF23 and cognitive function in hemodialysis patients [19]. In addition, VD deficiency is more common in the elderly population, and a variety of studies have indicated the interrelationship between VD and elderly cognitive function [20, 21]. Some studies have found that VD not only exhibits classical regulation of bone and calcium and phosphorus metabolism, but also shows immunomodulatory, anti-inflammatory, and antifibrotic effects [22].

The nuclear factor kappa-B (NF-*κ*B) signaling pathway is of vital significance in LOAD inflammatory response. When the brain tissue gets inflamed, it acts as a key mediator, stimulating microglia activation and amplifying the inflammatory response caused by internal and external factors [23, 24]. Won et al. have found that VD protects blood-brain barrier from hypoxia and reoxygenation damage by inhibiting activation of NF-*κ*B pathway as well as mediating inflammatory response [25]. Zhao et al. found that, in the blood of patients with diabetes mellitus, KL protein may reduce I-*κ*B phosphorylation by regulating I-*κ*B kinase (IKK). Therefore, the activation of NF-*κ*B signaling pathway was inhibited [26]. Furthermore, studies have shown that KL and VD are closely related to the NF-*κ*B signaling pathway, and they both have negative correlations [27–29]. However, the relationship between KL-FGF23-VD axis and NF-*κ*B signaling pathway and IKK has not been reported yet.

To sum up, this study was conducted based on the rat model of LOAD induced by A*β* combined with IBO, and the cultured A*β* microglia stimulated by the mixture of A*β* and IBO. And the relationship between KL-FGF23-VD axis and LOAD was explored. It is hypothesized that the KL-FGF23-VD axis can mediate NF-*κ*B signaling pathway activation via regulating IKK, inhibit the enhancement of inflammatory response of microglia, prevent neuron damage, and inhibit the progression of LOAD. The mechanism of neuroinflammation is explored through NF-*κ*B signaling pathway, which is expected to provide a new target for LOAD therapy.

## 2. Materials and Methods

### 2.1. A*β* Combined with IBO Inducing LOAD Rats

A total of 84 aged SD rats (18 months old, male, body weight 550 ± 50 g, SPF grade) were purchased from Chongqing Medical University. The animal experiments were carried out as per the protocols with approval of the First Affiliated Hospital of Chengdu Medical College. 12 rats were set as blank group (Control) without any intervention. The remaining 72 rats were divided into KL gene knockdown group (KL-si), KL gene enhancement group (KL-OE), and empty vector group (NC), with 24 rats in each (rats in KL-si group were transduced with KL gene interfering adenovirus; KL-OE group was transduced with adenovirus overexpressing KL gene; NC group was transduced with empty vector). The above three groups are then randomly divided into two subgroups with 12 rats in each subgroup. A subgroup (A*β*) was injected with 1.5 *μ*L of A*β*_1-40_ (HY–P0265; MedChemExpress) and IBO (A137136; Aladdin) mixture after localization of hippocampal CA1 region, and the other (NS) was injected with normal saline at the same site, and the operation steps were the same. In summary, all rats were divided into 7 groups, namely, Control group, KL-OE/A*β* group, KL-OE/NS group, KL-si/A*β* group, KL-si/NS group, NC/A*β* group, and NC/NS group. After anesthesia, the rats were located in the CA1 area (with the bregma point as the origin, the coordinates of the CA1 area in the hippocampus are AP3.6 mm, ML2.0 mm, DV3.0 mm) with brain stereotaxic instrument, and the virus was injected into the bilateral hippocampus with a volume of 1 *μ*L/site, and the speed was 0.2 *μ*L/min a micro-injection needle. After staying for 20 minutes, one subgroup was given 1.5 *μ*L of A*β*_1-40_ (10 g/L) and IBO (0.6 *μ*g/*μ*L) in the hippocampal CA1 area, while the other subgroup was injected with normal saline at the same area, and the needles were left for 5 minutes. The needles were withdrawn and sutured and then put back into the cage. Relevant tests continued after 10 days of continuous feeding. After the rat was anesthetized, the brain was cut open, and the rat brain tissue was taken out, rinsed in ice-cold saline, and dried with filter paper, and the brain was put on the ice table with ophthalmic forceps to quickly peel off the hippocampus, then temporarily store it in liquid nitrogen, and then transfer to a −80°C refrigerator for storage until subsequent experiments.

### 2.2. Isolation and Culture of Primary Microglia

Microglia from the hippocampus of rats' brain tissue were isolated and purified by primary isolation method. Cells were cultured in high glucose DMEM medium (11965092; ThermoFisherScientific) containing 1% penicillin-streptomycin (C0009; Beyotime) and 10% FBS (PS-FB5-SA; Peakserum) in a 37°C incubator with 5% CO_2_. The purified and cultured microglia were stimulated with the mixture of A*β* and IBO (referred to as A*β* microglia). The above cells were divided into 6 groups: KL overexpressing adenovirus transfected A*β* microglia (KL-OE); KL shRNA transfected A*β* microglia (KL-si); IKK-16 (a specific inhibitor of IKK) purchased from Selleck was added to A*β* microglia (IKK-16); KL overexpressing adenovirus was introduced into A*β* microglia, and then IKK-16 was added (KL-OE/IKK-16); empty vector was introduced into A*β* microglia (NC) and A*β* microglia (Control). After 48 h of adenovirus infection, IKK-16 (1 *μ*M) or the same amount of DMSO was pretreated for 30 min, and then A*β* (0.55 *μ*M) and IBO (0.6 *μ*M) were mixed for 48 h, and the cells were collected.

### 2.3. Histopathology

The brain tissue was embedded in paraffin, sliced, mounted, dehydrated in ethanol, stained with hematoxylin (G1004; Servicebio) and eosin (G1002; Servicebio), and cleared with xylene to make sections. The images of the slices were collected using the Mshot MF53 microscope (Guangzhou Mshot Photoelectronic Technology Co., Ltd.), and histopathological status was observed.

### 2.4. NF-*κ*B Fluorescent Staining

Followed by three cycles of washing with PBS, 5 min each, 0.5% TritonX-100 was provided dropwise to slides and let stand by for 10 min at room temperature. The slides were immersed in PBS 3 times, 3 min each, blocked by using 10% normal goat serum (C0265; Beyotime) at room temperature, and removed after blocking for 60 min. The primary antibody diluent (P0262; Beyotime) was supplemented, placed in a humid chamber, and incubated at 4°C overnight. The slides were rewarmed at room temperature for 30 min and soaked in PBS for 3 times, 3 min each. Excess liquid was removed, and fluorescent secondary antibody was diluted and added for incubation at 37 °C for 60 min. PBS immersion was conducted for 3 times again, 3 min each. Following the addition of DAPI (C1005; Beyotime), the cells were incubated in the dark for 5 min and stained for nucleus. Antifluorescence quenching medium was added to mount the slides, and the experimental results were collected using fluorescence microscope imaging system (MF53; Guangzhou Mshot Photoelectronic Technology Co., Ltd.).

### 2.5. Flow Cytometry

The flow cytometry was performed using Annexin V-APC/DAPI Apoptosis Kit as per manufacturer's instructions (E-CK-A258; Elabscience). After the experimental animals were anesthetized, the skull was opened to expose the brain, and the hippocampus was isolated and then put into in frozen PBS. The tissue was cut into small pieces of about 1 mm3, 0.25% trypsin (S310 KJ; Beyotime) was used for digestion at 37 °C for 20 min, and DMEM was provided to terminate the digestion. After being collected, the cell suspension was centrifuged at 1000 rpm for 5 min, added with PBS, and allowed to make a single cell suspension (4 × 10^5^ cells/mL), and we repeated centrifugation again at 300 g for 5 min, discarded the supernatant, resuspended cells and repeated again, then washed with PBS, and added 100 *μ*L diluted 1×Annexin V Binding Buffer to resuspend cells in solution. 2.5 *μ*L Annexin V-APC plus an equal quantity of DAPI staining solution was supplied, and the cell suspension was incubated in the dark at room temperature for 20 mi, added to 400 *μ*L diluted 1×Annexin V Binding Buffer, and detected in a flow cytometer CytoFLEX (Beckman, USA).

### 2.6. Transmission Electron Microscope

The tissue in the hippocampal CA1 area was quickly separated under stereo microscope within 1∼3 min after the animals were sacrificed, placed in the fixative solution on the wax slide, cut into tissue pieces of about 1 mm 3 size with a blade precooled at 4°C, and fixed with 4% glutaraldehyde for 2 h. After being washed 3 times with PBS, 10–15 min each time, the tissues were fixed using 1% osmium tetroxide for 2h. After PBS washing for three times, it was dehydrated twice with concentration gradient acetone, embedded by epoxy resin, and placed in an oven for polymerization. Then, the tissue was prepared into ultrathin slices with a thickness of 50 nm by using an ultramicrotome, stained in uranyl acetate and citric acid for 20 min at RT and observed using a transmission electron microscope (Hitachi H-7500; Hitachi Construction Machinery Co., Ltd.).

### 2.7. qPCR

The total RNA of hippocampus in rat brain was extracted using Trizol kit (15596026; ThermoFisherScientific). RNA reverse transcription was accomplished using Goldenstar RT6 cDNA Synthesis Mix Kit (Tsingke Biotechnology Co., Ltd.). First, a PCR reaction solution was prepared: 10 *μ*l of 2×T5 Fast qPCR Mix, 0.8 *μ*l of 10 *μ*M Primer F and 10 *μ*M Primer R, 0.5 *μ*l of Template DNA, 0.4 *μ*l of 50×ROX Reference Dye II, and dd H_2_O to make up the system to 20 *μ*l. The conditions for PCR reaction were 95°C for 5 s, 55 °C for 30 s, and 72 °C for 30 s, 40 cycles (See Table 1).

### 2.8. ELISA

ELISA assay was exploited to detect the levels of vitamin D in the hippocampus and cortex of the rat brain as per manufacturer's instructions (tw046046, Shanghai Tongwei Biotechnology Co., Ltd.). FGF23 (CEA746Ra) and APP (SEB020Ra), IL-1 (tw039546), IL-2 (tw039579), IL-6 (tw039608), TNF-*α* (TWp002859), and VD (tw046046) expression in microglial secretions were also detected by ELISA assay. ELISA kits of FGF23 (CEA746Ra) and APP were purchased from Cloud-clone Corp (Wuhan, China); IL-1, IL-2, IL-6, TNF-*α* and VD were in Shanghai Tongwei Biotechnology Co., Ltd.

### 2.9. Western Blotting

The protein was extracted by adding RIPA lysis buffer, vortex for 1 min, and then was placed on ice for 10 min, and this is repeated three times. Then, the mixture was centrifuged at 13000 rpm for 20 min at 4 °C, and the supernatant was collected. Protein was quantified by BCA, denaturation at 100°C for 6 min. After the proteins were separated with 13% SDS-polyacrylamide gel electrophoresis, they were transferred to a PVDF membrane and blocked using skim milk for 1 h. The membrane was cleaned with TBST for 3 times, each time for 5 min. Primary antibody (1 : 1000) was supplemented and cultured overnight at 4 °C. After TBST washing, secondary antibody (1 : 2000) was supplemented and incubated at 37 °C for 1 h. After TBST washing, chemiluminescence color was triggered, and the optical density of the band was analyzed. The bands were quantified by densitometry using Image J software, and *β*-Actin was used as the internal control. The primary antibodies were purchased from ABclonal: anti-KL (A12028), anti-FGF23 (A6124), anti-APP (A11019), anti-IL-1 (A1316), anti-IL-2 (A0302), anti-IL-6 (A0286), anti-TNF-*α* (A11534), anti-IKK (A2087), and anti-*β*-Actin (AC026).

### 2.10. Immunohistochemistry

After being paraffin-embedded, the tissues were prepared as 4 *µ*m thickness slices, deparaffinized, and dehydrated. By the addition of 3% hydrogen peroxide, the sections were cultured at room temperature for 15 min in the dark to block the action of endogenous peroxidase. The slices were washed 3 times with PBS and then blocked with goat serum for 60 min at room temperature. Following the removal of blocking solution, primary antibody (A0208; Beyotime) was added for incubation overnight at 4°C. One day after the PBS washing, the secondary antibody was supplied and incubated at room temperature for 1.5 h. After three cycles of PBS washing, fresh DAB was added and incubated in the dark for 10 min, and the color development was terminated by washing with water. Then, it was counterstained using hematoxylin for 5 min, cleaned using tap water until returned to blue, and finally dehydrated, permeabilized, and sealed with neutral gum. Images of the slices were collected using a Mshot MF53 inverted microscope produced by Guangzhou Mshot Photoelectronic Technology Co., Ltd. The secondary antibody A*β* pAb (A16265; ABclonal) and NF-*κ*B antibody (436700; ThermoFisherScientific) were purchased.

### 2.11. Statistical Analysis

All experiments were performed three times independently, and the collected data were expressed as mean ± standard deviation. GraphPad Prism version 9.0 (GraphPad Software; San Diego CA) was employed for statistical analysis. Multiple group comparison was employed using one-way analysis of variance (ANOVA) followed by a Tukey's post hoc test. The value of *P* less than 0.05 indicated that the difference was statistically significant.

## 3. Results

### 3.1. KL-FGF23-VD Axis Improves Inflammation and Reduces A*β* Accumulation in Brain

Immunohistochemical staining was used to detect the A*β* deposition in rat brain tissues. A*β* deposition was markedly elevated in the brain of A*β* combined with IBO induced LOAD rats compared with controls, and the number of brown positive cells was increased (Figure 1(a)). KL gene can reduce A*β* accumulation in the brain of LOAD rats that A*β* accumulation in KL-OE was decreased in contrast to KL-si and NC. By comparison with the control group, immunohistochemical detection of NF-*κ*B showed that NF-*κ*B expression was increased in the A*β* group; especially the NF-*κ*B positive cells in the KL-si/A*β* group were apparently aggregated (Figure 1(b)), while KL gene can inhibit NF-*κ*B expression that is decreased in KL-OE/A*β* compared with KL-si/A*β* and NC/A*β*. When the ultrastructure of hippocampal microglia was observed by electron microscope, it was found that microglia in the A*β* group were activated, and the lysosomes were increased (Figure 1(c)). The activation of hippocampal microglia in LOAD rats in the KL-OE group was inhibited, NF-*κ*B expression was decreased, inflammatory response was alleviated, and A*β* deposition in the brain was reduced (Figure 1).

HE staining was used to observe the inflammation of brain tissue and surrounding tissues in each group, and it was found that inflammatory cell infiltration, neuronal cell vacuolar degeneration, and damage deformation were found in the KL-si/A*β* group. The neuronal cells in the NC/A*β* group were loosely arranged, and the glial cells increased (Figure 2(a)). Inflammatory indexes IL-1, IL-2, IL-6, and TNF-*α* in rat brain were increased in KL-si/A*β* and NC/A*β* groups (Figure 2(b)). KL gene can improve the pathology of rat brain tissue and alleviate the surrounding inflammation. As shown in Figures 2(a) and 2(b), the histopathology was improved in the KL-OE group, and the inflammatory indexes were reduced, and the level of inflammatory factors in the KL-OE/A*β* group was comparable to the Control.

When the apoptosis of hippocampal neurons in each group was detected using flow cytometry, the number of apoptotic neurons in the A*β* group increased, and the KL-OE group was comparable to the control group in that KL gene could reduce the apoptosis of neurons in LOAD rats (Figure 2(c)). In addition, FGF23 participated in the regulation of VD metabolism, and decreased secretion of FGF23 led to increased production of VD. The roles of this axis in the gut, bone, thyroid, and kidney have been reported. Our study found that protein KL was enhanced after KL was overexpressed in rats, and KL could reduce FGF23 and APP expression in the brain tissue of LOAD rats, and that of the KL-OE/A*β* group was comparable to that of the control group (Figure 3(a)–3(d)). The transcriptional expression of KL gene in the brain hippocampus is shown in Figure 3(e), and the transcriptional expression of KL gene was increased after transduction of KL overexpressed gene. These findings suggest the potential participation of KL-FGF23-VD in alleviating the pathological conditions of brain tissue in LOAD rats, inhibiting NF-*κ*B pathway activation while improving brain tissue inflammation and clearing A*β* deposition.

### 3.2. KL-FGF23-VD Axis Inhibits NF-*κ*B Signaling Pathway and A*β* Microglia Activation by Regulating IKK

Microglia can activate and amplify NF-*κ*B signaling pathway that is essential in LOAD inflammatory response. In the microglia, which are stimulated by the mixture of A*β* and IBO, the cell ultrastructure was visualized using a transmission electron microscope. In A*β* microglia (Control group), the nucleus was deformed, mitochondria were swollen, and flocculent deformed, and multiple lysosomes were found. In the KL-OE and KL-OE/IKK-16 groups, the nucleus was round and plump, the chromatin was evenly distributed, and the subcellular structure was normal (Figure 4(a)). NF-*κ*B activation in microglial cells was detected using immunofluorescence. NF-*κ*B expression in the nucleus was evidently elevated in the KL-si group and decreased in the KL-OE and IKK-16 groups, and NF-*κ*B was almost not expressed in the cytoplasm and nucleus in KL-OE/IKK group (Figure 4(b)). After KL-OE treatment, KL gene transcription and protein expression were increased in A*β* microglia (Figures 5(a)–5(c)). In addition, Western blotting results revealed that, in A*β* microglia, IKK and NF-*κ*B expression were markedly increased in the KL-si group, and the expression levels were significantly decreased after KL-OE and IKK-16 treatment and further decreased in KL-OE/IKK-16 compared with KL-OE and IKK-16 (Figures 5(d) and 5(e)).

To further explore the effect of KL on inflammatory markers in A*β* microglia and the possible mechanism in the inhibition of NF-*κ*B pathway activation, we used ELISA to detect the levels of inflammatory markers IL-1, IL-2, IL-6, and TNF-*α* in A*β* microglia as well as the expression of FGF23-VD axis and APP protein. The levels of FGF23 and APP were substantially elevated in the KL-si group and decreased in the KL-OE, IKK-16, and KL-OE/IKK-16 groups (Figures 6(a)-6(b)). The previously described markers were largely increased in the KL-si group, while KL-OE and IKK-16 could reduce the inflammatory indicators (Figures 6(c)–6(f)). The correlation between VD and cognitive function in old age has been confirmed in some studies, and VD deficiency is considered to be one of the risk factors for LOAD. The levels of VD in A*β* microglia were increased in the KL-OE, IKK-16, and KL-OE/IKK-16 groups. After knockdown of the KL gene, the metabolism of VD in the KL-si group decreased, and the KL gene could increase the metabolism of VD in A*β* microglia (Figure 6(g)).

## 4. Discussion

AD is divided into early-onset and late-onset AD. More than 95% of patients are classified as LOAD, which is different from early-onset dominant genetic diseases and is a multifactorial disease and easily susceptible to living environment and lifestyle [30]. AD has an insidious onset, and a slow course of disease, and is often accompanied by progressive memory impairment, cognitive dysfunction, and emotional dysfunction. As one of the most common diseases in senile dementia, it is also known as senile dementia [31]. AD can be divided into three stages, that is, mild, moderate, and severe, according to the clinical course of the patient. The mild patients have impaired calculation and memory skills and attention deficits. In severe patients, they will lose behavior ability, cannot take care of themselves, lose language skills, and rely on the care of others to survive, which poses a great threat to the patient's life and health [32].

The KL gene can be antiaging, and it is related to human later life and central nervous function, possessing the effect of protecting hippocampal neurons. In addition, studies have found that KL in plasma is correlated with cognitive function of the elderly without dementia. KL gene improves cognition and reduces mortality in mice with dementia. FGF23 is an endocrine factor secreted by osteoblasts, which is relevant in regulating VD metabolism in the body. The KL protein can block the expression of FGF23, and the study found that the secretion of FGF23 protein increased in KL knockout mice. Kosakai et al. found that the expression of VD was abnormal in KL-deficient mice, suggesting that KL and VD are related and play a role in neurodegenerative diseases [33]. In recent years, Mohammadi used X-ray crystallographic analysis to induce the precipitation of FGF23 together with its receptor (FGFR) and KL protein from solution and form stacks of repetitive and ordered crystals, from which he considered FGF23 to be employed as a complex [34]. The increasing evidence has proved an intrinsic link between KL, FGF23, and VD, forming an endocrine axis that was reported in the gut, bone, thyroid, and kidney [35].

However, whether the KL-FGF23-VD axis is vital in the treatment of LOAD disease has not yet been reported. Therefore, we designed experiments to explore the protective effect of KL-FGF23-VD axis in LOAD model rats and microglia through animal and cell experiments using the silencing and enhancement of KL gene. In the LOAD rats, we found that, unlike KL-si that promotes aggravated brain tissue damage, promotes neuronal apoptosis and microglia activation, and aggravates tissue inflammation, enhanced KL expression (KL-OE) can reduce A*β* deposition, neuronal apoptosis in LOAD model rats, and inhibit microglial activation and inflammatory response in brain tissues. Zeng et al. found that aging mice with early renal insufficiency had increased TNF-*α*, IL-1, etc., decreased KL protein, and increased activation of NF-*κ*B signaling pathway [36]. Intracranial KL protein decreased, and NF-*κ*B pathway activation was increased in hippocampus and frontal cortex, and inflammatory indicators such as IL-1, TNF-*α*, and IL-6 in nephrectomized mice with cognitive impairment, suggesting that KL protein and NF-*κ*B signaling pathway are negatively correlated [37]. In addition, the activation of microglia has been reported to be related to the activation of NF-*κ*B. Our results showed that, in KL-OE group, the transcription level of KL gene in the hippocampus was elevated, the inflammatory indicators IL-1, TNF-*α*, and IL-6 were decreased, and the NF-*κ*B pathway and microglial activation were inhibited. KL, FGF23 and VD are secreted in human cerebrospinal fluid and blood [38]. Studies have revealed that patients with multiple sclerosis had increased FGF23 and phosphorus levels in cerebrospinal fluid than normal people, and KL protein, VD, and calcium ions decreased. It is suggested that, in the inflammatory environment, the KL-FGF23-VD axis plays an anti-inflammatory role, and the decrease of VD and calcium ions reduces the neuroprotective effect [18]. When we detected the expression of KL-FGF23-VD axis protein in the LOAD hippocampus by WB, we found that FGF23 was decreased in the KL-OE group. The results indicated that the KL-FGF23-VD axis was involved in reducing the A*β* deposition in the brain of LOAD rats, alleviating the neuronal cell damage, and mediating both NF-*κ*B and microglial activation.

In order to further explore that KL-FGF23-VD axis inhibits the NF-*κ*B signaling pathway activation via the action on IKK, a rate-limiting enzyme, thereby reducing the microglial activation and the degree of inflammatory response of microglia in LOAD, we stimulated the purified and cultured microglia with the mixture of A*β* and IBO and added IKK-16, a specific inhibitor of IKK, to investigate the regulatory effect of KL-FGF23-VD on IKK. Consistent with animal experiments, KL gene transcription and protein levels were increased in A*β* microglia KL-OE group, FGF23 was decreased, and VD expression was increased. A global expert consensus in Boston identified VD deficiency as a risk factor for LOAD in 2003 [20]. Among other neurodegenerative diseases, namely, Parkinson's disease, Calvello found that VD plays a neuroprotective role in Parkinson's disease patients, and it exerts an effect by mediating proinflammatory and anti-inflammatory factors [39]. After adding IKK-16 to the KL-OE group, compared with the KL-OE and IKK groups, FGF23 protein expression was decreased, while KL and VD were increased. It was also found that the expression of IKK in KL-si microglia was significantly increased, and KL-OE and IKK-16 could reduce the expression of IKK in A*β* microglia, especially in the KL-OE/IKK-16 group. These results suggested that the KL-FGF23-VD axis can regulate the expression of IKK in A*β* microglia. In addition, KL-OE can reduce the secretion of the inflammatory factors in A*β* microglia in the previously described. In resting cells, NF-*κ*B and its inhibitor of nuclear factor-*κ*B (I-*κ*B) exist in the cytoplasm as an inactive dimer (NF-*κ*B-I-*κ*B). In response to external signals, IKK promotes the phosphorylation of I-*κ*B, NF-*κ*B is separated from I-*κ*B, and NF-*κ*B is activated and transferred into the nucleus, where it quickly associates with the corresponding NF-*κ*B binding sites on target genes interaction to regulate target gene expression (producing cellular responses such as inflammation and immunity) [40]. The effect of KL-FGF23-VD axis on NF-*κ*B signaling and microglia activation was further explored by fluorescence staining and transmission electron microscopy, and the results showed that NF-*κ*B signaling was abundantly expressed in the nucleus in the KL-si group and significantly decreased in the KL-OE and IKK-16 group, while there is almost no expression in the cytoplasm and nucleus of the KL-OE/IKK-16 group, indicating that microglia and NF-*κ*B signaling activation are suppressed in KL-OE, IKK-16, and KL-OE/IKK-16 groups. The results proved that KL-FGF23-VD axis can inhibit NF-*κ*B signaling and activation of microglia by regulating IKK and reduce the degree of inflammatory response of microglia.

## 5. Conclusions

The present study indicates a potential regulation role of KL-FGF23-VD axis in attenuating brain inflammation and inhibiting neuronal apoptosis and microglia activation in AD, which may be effective by regulating IKK/NF-*κ*B signal pathway.

## Figures and Tables

**Figure 1:** A*β* accumulation in brain was detected by Immunohistochemical staining. (a) Immunohistochemical staining of A*β* deposition in the brain of rats (*n* = 3). (b) Immunohistochemical staining of NF-*κ*B expression in hippocampus of rats (*n* = 3). The nucleus was in blue and the positive A*β* and NF-*κ*B cells were colored in brown. Scale bar = 50 *µ*m. (c) Ultrastructure of rats' hippocampal microglia (*n* = 2).

**Figure 2:** The nerve protective role of KL gene in LOAD rats. (a) HE staining of rats brain (*n* = 3). Scale bar = 50 *µ*m. (b) Expression of IL-1, IL-2, IL-6, and TNF-*α* in rat hippocampus was detected using Western blot, semiquantitative analysis was employed based on *β*-actin (*n* = 3). (c) Apoptotic neurons in each group (*n* = 3). One-way ANOVA assay was used for pairwise comparison. ##*P* < 0.01, compared with control.

**Figure 3:** KL gene deceases FGF23 expression. (a) Expression of KL, FGF23, and APP in hippocampus of rats was detected using Western blot (*n* = 3). The semiquantitative analysis of protein KL (b), FGF23 (c), and APP (d) was employed based on *β*-actin. (E) KL gene expression in hippocampus of rats (*n* = 3). One-way ANOVA assay was used to for pairwise comparison. ##*P* < 0.01, compared with control.

**Figure 4:** KL gene inhibits A*β* microglia activation. (a) Ultrastructure of A*β* microglia. (b) Expression of NF-*κ*B in A*β* microglia was detected by Immunofluorescence staining. Scale bar = 50 *µ*m.

**Figure 5:** Expression of KL, NF-*κ*B, and IKK in microglia. (a) KL gene expression in microglia. (b) KL, NF-*κ*B, and IKK protein expression in microglia. The quantitative analysis of protein KL (c), NF-*κ*B (d), and IKK (e) was shown. One-way ANOVA assay was used for pairwise comparison. #*P* < 0.05, ##*P* < 0.01 vs control.

**Figure 6:** Contents of (a) FGF23, (b) APP, (c) IL-1, (d) IL-2, (e) IL-6, (f) TNF-*α,* and (g) VD in microglial secretions. One-way ANOVA assay was used for pairwise comparison. ##*P* < 0.01, compared with control.

**Table 1:** Primers used in RT-qPCR.

KL-F	5'-CGACAGTTACAACAACGTCTAC-3'
KL-R	5'-CACGATATGGAGAAGCGGTAG-3'
GAPDH-F	5'-GCAAGTTCAACGGCACAG-3'
GAPDH-R	5'-GCCAGTAGACTCCACGACATA-3'

## Data Availability

The data used to support the findings of this study are included within the article. The raw data has been uploaded to the following link: https://www.jianguoyun.com/p/DVlm4Z0Q3JuIChiTgL8EIAA.
